The article "Investigation of the Correlation between Cuff Inflatable Hypertension and the Difference in Interarm Diastolic Pressure Induced by Single Arm Ischemia" was published in 2022. Journal: Contrast Media Mol Imaging.

# Investigation of the Correlation between Cuff Inflatable Hypertension and the Difference in Interarm Diastolic Pressure Induced by Single Arm Ischemia

**DOI:** 10.1155/2022/9796737

**Published:** 2022-09-28

**Authors:** Yi Li, Wen Zhong, Weitong Hu, Liang Zhou, Renhong Wang, Meizhen Xu

**Affiliations:** ^1^Department of Cardiac Intervention, The Second Affiliated Hospital of Nanchang University, Nanchang 330006, China; ^2^Department of Cardiology, The Second Affiliated Hospital of Nanchang University, Nanchang 330006, China

## Abstract

The correlation between cuff inflatable hypertension and the difference in interarm diastolic pressure induced by single arm ischemia is investigated. A total of 126 patients undergoing coronary angiography in our hospital from January 2020 to January 2021 are selected and divided into the non-pseudohypertension (non-PHT) group (64 cases) and the PHT group (62 cases) according to the difference between systolic blood pressure and diastolic blood pressure measured directly and indirectly. The patients are subjected to the beam arm ischemia test and blood pressure measurement. The diastolic pressure differences between the patients before and after the beam arm are analyzed, and endothelial function and imaging indicators are compared. The risk factors for PHT are analyzed by binary logistic regression, and the diagnostic efficacy of diastolic blood pressure difference interarms (DBPI-r) for PHT patients is analyzed by receiver operating characteristic (ROC) curve. The experimental results show that the diastolic pressure difference induced by single arm ischemia can be used in the diagnosis of cuff inflatable hypertension.

## 1. Introduction

Hypertension is a relatively common chronic disease with a high prevalence and easy to induce cardiovascular and cerebrovascular diseases [1, 2]. Pseudohypertension (PHT) is a condition in which blood pressure measured through a cuff is not true and blood pressure is higher than that measured directly through an arterial puncture. Cuff inflatable hypertension is a relatively rare condition in PHT, which only occurs in a small number of people. The reason may be that some people are sensitive to cuff inflatable, which leads to a significant increase in blood pressure, resulting in significant measurement error and affecting diagnosis results [3]. The cuff inflatable hypertension patients for routine hypertension treatment may make not only patients excessive blood pressure but also may damage the health of patients. Yue et al. showed that the mechanism of pseudohypertension may be related to local arteriosclerosis, or it may be caused by abnormal nerve mediating after inflating the cuff, which leads to increased blood pressure [4]. At present, an invasive blood pressure test is more commonly used in clinical diagnosis of PHT, and the test results are relatively accurate [5]. However, this method has some disadvantages. The catheter is inserted into the artery and the pressure probe is used to measure the intracavity pressure, which is invasive and not well accepted by patients. Noninvasive methods such as pulse wave velocity (PWV) and flow mediated dilatation (FMD) can also play a good diagnostic effect on PHT, but this method has certain requirements on the professionalism of the examiners. Related equipment and materials are expensive, so it is difficult to be widely applied in clinical practice [6, 7].

The article "Investigation of the Correlation between Cuff Inflatable Hypertension and the Difference in Interarm Diastolic Pressure Induced by Single Arm Ischemia" was published in 2022. Journal: Contrast Media Mol Imaging.

At present, there is still a lack of good noninvasive detection methods for clinical diagnosis of PHT. Studies have shown that the beam arm ischemia test is a good way to test vascular endothelial function, and the degree of arterial stiffness can also be detected [8]. The cuff arm ischemia experiment is performed on the patient. The patient's arm is bound with a cuff, and the cuff is inflated to compress the brachial artery of the patient for 5 minutes; then, the cuff is deflated. Therefore, isometric diastolic pressure may be a new noninvasive method to diagnose cuff inflatable hypertension. Therefore, this study aims to explore and analyze the correlation between cuff inflatable hypertension and the difference in interarm relaxation induced by single-arm ischemia, so as to provide more reference for clinical application.

The rest of this study is organized as follows: Section 2 discusses related work, followed by general information and detailed methods designed in Section 3.  Section 4 shows the experimental results, and Section 5 concludes the study with summary and future research directions.

## 2. Related Work

PHT referred to actual normal blood pressure, which was caused by local arterial stiffness or neuromediated pressure, resulting in the illusion of elevated blood pressure during detection [9]. Among them, the specific mechanism of cuff inflatable hypertension is unknown, but it was believed that it has a similar physiological basis to hypertension. Invasive blood pressure testing was the preferred method for diagnosing PHT in clinical practice, which was more accurate, but difficult to be widely used in clinical screening due to its trauma [10]. In addition, noninvasive methods such as PWV and FMD can also be used to diagnose PHT, but these methods have high requirements on testing personnel and equipment and were also difficult to be widely applied in clinical practice [11]. At present, there was still a lack of reliable noninvasive methods to diagnose PHT in the clinic. Studies have found that the brachial ischemia test has a good effect on the detection of vascular endothelial function, and this method can change the diastolic blood pressure between the arms of patients, which was similar to the principle of FMD, that is, reactive congestion increases shear forces, promotes the release of endogenous nitric oxide (NO) by blood vessels, dilates blood vessels, and leads to a drop in blood pressure [12]. Endothelin (ET) and vascular endothelial active peptide NO can be tested by this method, which can be used to determine vascular endothelial function. The research team led by Kim et al. [13] showed that the levels of ET and NO in patients with hypertension and coronary heart disease were abnormal, usually manifested as high ET levels and low NO levels. This study showed that cuff inflatable hypertension was correlated with the difference in interarm relaxation induced by single-arm ischemia, and the difference in interarm relaxation induced by single-arm ischemia could be used to judge cuff inflatable hypertension.

The article "Investigation of the Correlation between Cuff Inflatable Hypertension and the Difference in Interarm Diastolic Pressure Induced by Single Arm Ischemia" was published in 2022. Journal: Contrast Media Mol Imaging.

Domestic research studies by Fan et al. [14] showed that FMD can diagnose vascular endothelia, indicate NO concentration level, and reflect arterial vasodilation, which was similar to the results of this study. The results of this study showed that compared with the non-PHT group, the posterior interbrachial of the PHT group was smaller, *P* < 0.05. An analysis of its mechanism was that patients with cuff hypertension have lower interbrachial diastolic pressure, which may be caused by impaired endothelial function. The principle of interbrachial diastolic pressure behind the banding arm was similar to that of FMD. The lower interbrachial diastolic pressure indicates poor vascular elasticity and impaired endothelial function. A higher interarm diastolic pressure indicates better elasticity [15].

It was found that there were no significant differences in the data of left ventricular end-systolic diameter, left ventricular end-diastolic diameter, septal thickness, and carotid artery intima thickness (*P* > 0.05). Compared with the non-PHT group, the PHT group had more patients with left ventricular diastolic dysfunction, accounting for 70.97% (*P* < 0.05). Analysis of the reason is that in patients with hypertension with cuff inflatable cuff, a one-arm ischemia test will cause increased blood pressure and abnormal hemodynamics, thus affecting endothelial function and arterial vascular dilation, resulting in small differences in diastolic blood pressure between arms, thus weakening left ventricular diastolic function. This is similar to the research results of Xu et al. [16]. In this study, diastolic pressure changes after beam arm ischemia were not very significant in the PHT group, which may be related to the vascular endothelial function of the body. Binary logistic regression analysis showed that DBPI-r behind the beam arm, ET before the beam arm, and ET behind the beam arm were independent risk factors for PHT. ROC curve was used to analyze the diagnostic efficiency of DBPI-r for PHT after the beam arm. It was found that DBPI-r has high diagnostic efficiency in PHT occurrence, and the beam arm test was simple to operate and less affected by other factors, which was easy to be accepted by patients. Therefore, DBPI-r can be popularized to screen PHT patients.

The article "Investigation of the Correlation between Cuff Inflatable Hypertension and the Difference in Interarm Diastolic Pressure Induced by Single Arm Ischemia" was published in 2022. Journal: Contrast Media Mol Imaging.

Currently, FMD and PWV are the most commonly used noninvasive blood pressure tests to diagnose PHT. Compared with these two methods, the diastolic blood pressure difference induced by single arm ischemia can become a new noninvasive blood pressure detection method, which is not only simple, convenient, and easy to operate but also requires less technical personnel. The noninvasive detection method can greatly improve the acceptance ability of patients, which is conducive to the diagnosis of cuff hypertension. There are also shortcomings in this study. The sample size of this study is small and cannot represent all patients with cuff inflatable hypertension. Therefore, further research is needed to expand the sample size in the future.

## 3. General Information and Detailed Methods

### 3.1. General Information

A total of 126 patients who underwent coronary angiography in our hospital from January 2020 to January 2021 are selected according to the diagnostic criteria of PHT (systolic or diastolic blood pressure difference >10 mmHg), and the patients are divided into the non-PHT group (64 cases) and the PHT group (62 cases). The mean age of the PHT group is (56.32 ± 6.45) years old, with 33 males and 29 females. The mean age of the non-PHT group is (58.97 ± 7.28) years, with 34 males and 30 females. There are no significant differences in baseline data such as age and gender between the 2 groups (*P* > 0.05).

### 3.2. Detailed Methods

Instruments and equipment: Omron sphygmomanometer (German HEM-7330), mercury sphygmomanometer, pressure sensor, ECG monitor, ET kit, NO kit, and ONOO kit.

The experimental procedure of bundle arm ischemia is performed on the patients [17]. The specific contents are as follows: before the measurement, the patients are required to empty the bladder, rest in a quiet and comfortable environment for 10–15 min, and take the decubitus position when the blood pressure is measured, with the sleeves rolled up and arms exposed. Two Omron sphygmomanometers of the same model are used to measure the patients' bilateral upper arm blood pressure once every 1 min, for a total of 3 times, to obtain the 3 blood pressure measurements and the average value [18, 19]. After the basic data of interarm blood pressure differences are obtained, a relatively narrow sphygmomanometer cuff is used to fix the patient's right upper arm, and the air is inflated to more than 40 mmHg above the patient's systolic blood pressure, so that the brachial artery blood flow is blocked for about 5 minutes, and then, the patient is quickly deflated. The blood pressure of both arms is measured at 1 min, 3 min, and 5 min after ventilation, and the difference between interarm systolic pressure and interarm diastolic pressure after one-arm ischemia is calculated at 1 min, 3 min, and 5 min.

The article "Investigation of the Correlation between Cuff Inflatable Hypertension and the Difference in Interarm Diastolic Pressure Induced by Single Arm Ischemia" was published in 2022. Journal: Contrast Media Mol Imaging.

An invasive blood pressure test is performed on the patient [20, 21], with the following details: 8 ml arterial blood is collected from the brachial artery of the patient's right hand using an angiographic catheter; a mercury sphygmomanometer is used to continuously inflate and pressurize the patient's right upper arm until it is higher than the patient's systolic blood pressure of 40 mmHg, maintained for 5 min, and 8 mL arterial blood is collected from the right brachial artery of the patient; and the collected arterial blood is centrifuged, and the concentration of ONOO-, NO, and ET in blood is detected.

### 3.3. Observation Indicators and Evaluation Criteria

The observed indicators of this study are as follows:

1. SBPI-r and DBPI-r differences before and after single-arm ischemia
2. Differences in endothelial function-related indicators
3. Differences in imaging indicators
4. Binary logistic regression analysis of risk factors for PHT
5. Analyze the utility of DBPI-r in clinical diagnosis of PHT after beam arm

### 3.4. Statistical Processing

The data in this study are processed by SPSS 26.0 software [22, 23]. All measurement data involved in this study are presented in the form of mean ± standard deviation $\left(\bar{x}\pm s\right)$, and a *t*-test is adopted. The statistical data are expressed in percentage (%), the *x*^*2*^ test is used, binary logistic regression is used to analyze the risk factors affecting PHT, and ROC curve is used to plot the diagnostic efficiency, if *P* < 0.05 proved to be statistically significant.

## 4. Experimental Results

### 4.1. Comparison of SBPI-r and DBPI-r between the Two Groups before and after Single-Arm Ischemia

Table 1 provides the differences in SBPI-r levels at different times. In Table 1, SBPI-r is the systolic blood pressure difference between arms (left arm SBP-right arm SBP).  Table 2 provides the differences in DBPI-r levels at different times. In Table 2, DBPI-r is a diastolic pressure difference between arms (left arm DBP-right arm DBP); “*a*” represents *P* < 0.05 compared to baseline; “*b*” represents *P* < 0.05 compared with the non-PHT group. Through the above experimental results, it can be observed that there is no significant difference in SBPI-r and DBPI-r levels at baseline and no significant difference in SBPI-r levels after single-arm ischemia (*P* > 0.05). After single-arm ischemia, DBPI-r is significantly increased, and compared with the non-PHT group, DBPI-R in the PHT group is lower.

The article "Investigation of the Correlation between Cuff Inflatable Hypertension and the Difference in Interarm Diastolic Pressure Induced by Single Arm Ischemia" was published in 2022. Journal: Contrast Media Mol Imaging.

### 4.2. Comparison of Endothelial Function-Related Indicators

Table 3 provides the comparison of endothelial function-related indicators. In Table 3, “*a*” stands for *P* < 0.05 compared with before beam arms of the same group; “*b*” stands for comparison between groups, *P* < 0.05. It can be seen from Table 3 that compared with the non-PHT group, the serum NO level in the PHT group is lower before and after beam arm (*P* < 0.05). ET level in the PHT group increased significantly than in the non-PHT group before and after beam arm (*P* < 0.05).

### 4.3. Comparison of the Differences of Imaging Indicators

Table 4 provides the comparison of imaging indicators. It can be seen from Table 4 that compared with the non-PHT group, there are more patients with left ventricular diastolic dysfunction in the PHT group (70.97%), *P* < 0.05.

### 4.4. Binary Logistic Regression Analysis of Risk Factors for PHT

According to the above statistical analysis results, indicators with *P* < 0.05 are included as independent variables, including DBPI-r behind the beam arm, NO before the beam arm, NO after the beam arm, ET before the beam arm, and ET after the beam arm.  Table 5 provides the risk factors for PHT by binary logistic regression analysis. It can be seen from Table 5 that DBPI-r behind the beam arm, ET before the beam arm, and ET after the beam arm are independent risk factors for PHT.

### 4.5. Analyse the Utility of DBPI-r in Clinical Diagnosis of PHT after Beam Arm

ROC curve is applied to analyze the utility of DBPI-r in diagnosing PHT behind the arm.  Figure 1 shows the ROC diagram of DBPI-r in diagnosing PHT patients. It is can be seen from Figure 1 that the area under the curve is high (AUC = 0.849), and the Yuden index is 0.68. When DBPI-r<3.5 mmHg, the optimal diagnostic cutoff value is 82.5%, and the specificity is 71%.

## 5. Conclusion

The correlation between cuff inflatable hypertension and the difference in interarm diastolic pressure induced by single arm ischemia is investigated. The diastolic pressure difference induced by single arm ischemia can be used to evaluate cuff inflatable hypertension. It is simple and noninvasive and can be a simple and effective indicator for cuff inflatable hypertension. The results of the study can be applied in clinical diagnosis, which can greatly enhance the identification and screening of PHT and reduce the occurrence of diagnostic errors.

The article "Investigation of the Correlation between Cuff Inflatable Hypertension and the Difference in Interarm Diastolic Pressure Induced by Single Arm Ischemia" was published in 2022. Journal: Contrast Media Mol Imaging.

## Figures and Tables

**Figure 1:** ROC diagram of DBPI-r in diagnosing PHT patients.

**Table 1:** Differences in SBPI-r levels at different times $\left(\bar{x}\pm s\right)$.

	SBPI-r	
	Non-PHT group	PHT group
The baseline	−0.83 ± 3.91	−0.91 ± 4.21
1 min	−0.98 ± 11.88	−0.32 ± 12.42
3 min	−0.59 ± 5.35	−0.35 ± 5.23
5 min	−0.51 ± 6.24	−0.26 ± 5.36

**Table 2:** Differences in DBPI-r levels at different times $\left(\bar{x}\pm s\right)$.

	DBPI-r	
	Non-PHT group	PHT group
The baseline	−1.25 ± 2.12	−0.32 ± 2.98
1 min	7.01 ± 3.46^a^	2.34 ± 3.77^ab^
3 min	5.31 ± 3.25^a^	1.96 ± 4.21^ab^
5 min	3.67 ± 3.78^a^	1.19 ± 3.68^ab^

a represents *P* < 0.05 compared to baseline; b represents *P* < 0.05 compared with the non-PHT group.

**Table 3:** Comparison of endothelial function-related indicators $\left(\bar{x}\pm s\right)$.

Indicators		Non-PHT group (*n* = 64)	PHT group (*n* = 62)
ONOO- (ng·L^−1^)	Before the beam of the arm	52.33 ± 3.23	50.43 ± 2.36
	After the beam of the arm	52.45 ± 3.36^a^	50.44 ± 2.19

ET (pg·L^−1^)	Before the beam of the arm	104.87 ± 10.89	112.26 ± 8.77^b^
	After the beam of the arm	106.02 ± 10.92^a^	113.35 ± 8.56^ab^

NO (ng·L^−1^)	Before the beam of the arm	117.19 ± 6.51	112.18 ± 6.36^b^
	After the beam of the arm	119.01 ± 7.53^a^	112.56 ± 8.77^ab^

a stands for *P* < 0.05 compared with before beam arms of the same group; b stands for comparison between groups, *P* < 0.05.

**Table 4:** Comparison of imaging indicators $\left(\bar{x}\pm s\right)$.

Indicators	Non-PHT group (*n* = 64)	PHT group (*n* = 62)	*P*
Left ventricular end contractile diameter (mm)	29.87 ± 4.26	32.38 ± 4.35	0.112
End diastolic diameter of the left ventricular (mm)	45.13 ± 4.38	47.72 ± 4.43	0.121
Interventricular septal thickness (mm)	9.55 ± 1.32	10.56 ± 1.74	0.139
Decreased left ventricular diastolic function (*n*, %)	25 (39.06%)	44 (70.97%)	0.028
Carotid intima-media thickness (mm)	0.88 ± 0.31	1.01 ± 0.19	0.119

**Table 5:** Risk factors for PHT by binary logistic regression analysis.

Indicators	*B*	Wald	*P*	EX (*B*)	95% CI
After the beam of the arm DBPI-r	−0.712	2.439	0.035	0.516	0.304–1.235
Before the beam of the arm ET	1.784	4.917	0.014	4.172	1.817–16.095
After the beam of the arm ET	1.815	5.036	0.021	0.408	0.094–0.947

## Data Availability

The data used to support the findings of this study are available from the corresponding author upon request.
